This article has been retracted.

# First Record of Ichthyofauna from Gomal Zam Dam, District South Waziristan, Khyber Pakhtunkhwa, Pakistan

**DOI:** 10.1155/2022/7076508

**Published:** 2022-11-19

**Authors:** Aziz Ur Rehman, Sami Ullah, Amina Zuberi, Farman Ullah Dawar, Muhammad Nasir Khan Khattak

**Affiliations:** ^1^Department of Zoology, Hazara University Mansehra, Khyber Pakhtunkhwa, Pakistan; ^2^Department of Animal Sciences, Quaid E Azam University, Islamabad, Pakistan; ^3^Department of Zoology, Kohat University of Science and Technology (KUST) Kohat, 26000 Khyber Pakhtunkhwa, Pakistan; ^4^Department of Applied Biology, College of Sciences, University of Sharjah, Sharjah, UAE

## Abstract

The present study reports the fish fauna of Gomal Zam Dam at three different sites from October 2018 to July 2019. The total sampled fish belong to 18 species, 15 genera, 5 families, and 4 orders. Fourteen species belong to family Cyprinidae, which was the most abundant, while one species belong to each family Mastacembelidae, Channidae, Siluridae, and Sisoridae. The prominent species were *Labeo dyochielus* (18.6%), *Barilius vagra* (16.5%), and *Barilius pakistanicus* (13.8%), while the rare species were *Tor zhobensis*, *Wallago attu*, *Hyphophthalmicthys molitrix*, *Ctenophyrngodon idella*, and *Bagarius bagarius* each one forming (0.1%). Species were rich in spring with ideal temperature, followed by summer, whereas species abundance was high in summer with high temperature and minimum abundance was recorded in autumn. In conclusion, the Gomal Zam Dam is a favorable reservoir for the fish particularly for family Cyprinidae. This present study will provide useful information about the diversity of fish fauna of Gomal Zam Dam that could be used in systematic fisheries management and conservation of the country.

## 1. Introduction

Fish are an essential human food source, rich in protein, fats, vitamins, phosphorus, and other fundamental elements. Fish live in diverse habitats and are found from the Arctic to the Antarctic zone of the world [1, 2]. Fish are distributed in nearly all natural aquatic environments, from colder to warmer. Based on feeding habits and other ecological factors, fish that live in warmer climates with relatively stable temperatures are abundant by species count [3]. The rich taxonomic and functional diversity of freshwater fish is due to their habitat isolation [4]. Thus, the rich biodiversity of freshwater ecosystems is the freshwater fishes [5]. Glaciated regions have fewer fish fauna than temperate regions [6]. More than 27,977 species comprise 62 orders and 515 families, with 450 families of freshwater fishes identified worldwide [7].

Pakistan has diverse fish fauna due to its biogeographical location, diversified agroclimatic conditions, and diverse eco- and geodiversity. Pakistan covered a total area of 780,000 hectares with a total wetland area of 9.7%, of which 73% is covered by freshwater and 26.06% is by coastal wetlands [8, 9]. The country has 193 species of freshwater, mainly belonging to the class Actinopterygii, subclass Teleostei [10, 11]. Studies examined the biodiversity of fish species in various water bodies in Khyber Pakhtunkhwa province of Pakistan, including River Kurram at Bannu [10–12] and Baran dam of district Bannu [13]. Khan et al. [14] recently determined the fish biodiversity of River Panjkora in both upper and lower Dir districts [14]. Ali et al. [15] studied the diversity of freshwater fishes from different locations of district Malakand including the Meherdi stream, Kharki stream, Wartier stream, Mahajar camp stream, and Dargai streams. According to Rafique and Khan [11], there are 193 freshwater fish species in Pakistan, including 5 superorders, 10 orders, 26 families, and 86 genera. The fish biodiversity from River Barandu, Pakistan was studied, and 18 species were identified [16].

The Gomal Zam Dam is constructed on river Gomal, originating from Afghanistan, and River Zhob emerging from Baluchistan, industrial-free areas; hence, the biodiversity of the Dam is conserved. Therefore, this study explored the ichthyofauna of the Gomal Zam Dam at three different sites and determined the physicochemical parameters of water. This study is the first-ever effort to record this newly constructed dam's fish fauna. Thus, the study will be attractive to Pakistan's fisheries sector and will add new understandings to the global fish industry.

## 2. Materials and Methods

### 2.1. Study Area

Gomal Zam Dam lies at 32°05′55^″^N and 69°52′53^″^E coordinates and is situated at Khajuri Katch of district South Waziristan, Khyber Pakhtunkhwa, Pakistan [17]. This dam impounds River Gomal, which emerges from Ghazni, Afghanistan and River Zhob, which emerges from Balochistan. The dam has been built for hydroelectric power generation, flood control, irrigation, and fish cultivation [18].

### 2.2. Study Design

The present study was carried out from October 2018 to July 2019 (10:00 am to 4:00 pm) and covered all the year's four seasons. Fish were sampled from three sites of the Dam (indicated in the map): Swai Nallah, Dotani village, and Gomal Khulla (Figure 1). Our previous protocol [16] was followed for fish and water sample collection. Sampling was carried out fortnightly from each site with the help of local fishermen where they have used gill nets with a length (10 m to 20 m), height (1.6 m), and mesh size of around 1.5 inches. Other nets like cast nets, drag nets, hand nets, and hooks were also used wherever necessary.

Similarly, water samples were collected from each site to determine its physicochemical parameters. Each catch was handled separately, and the specimens were sorted species-wise. The fish were preserved in 5-10% formalin for further identification in plastic jars. Small-sized fishes were immediately placed in the formalin solution, whereas formalin injection was given into the bodies of large-sized fishes before they were preserved in the formalin solution. The collection date, locality, and serial numbers were given to each collected and fixed fish species before they were saved in the laboratories of Fisheries and Aquaculture, Department of Animal Sciences, Quaid-I-Azam University Islamabad.

### 2.3. Fish Identification

The identification of the fish species was done mainly based on the color pattern, specific spots or marks on the body's surface, shape of the body, structure of various fins, and mouth shape. Identification was made after consulting several standard keys and literature, such as fishes of Punjab [19], freshwater fishes of the Indian region [20], and Pakistan May Taza Pane Ke Machlian [21]. During identification, different materials were used, such as surgical gloves, China dish, forceps for holding fish, measuring tape, facial masks, and a digital camera for capturing fish pictures.

### 2.4. Indices Used to Determine the Diversity

The following diversity indices were used to find fish species diversity.

### 2.5. Simpson's Index of Diversity (*D*)

(1) $$\begin{array}{c} D=1-\Sigma \left(pi2\right) \end{array}$$

Here, *pi* = *ni*/*N*, where *ni* is the total no. of individuals of a particular species and *N* is the total no. of individuals of all species. *Σ* = sum.

### 2.6. Pielou's Evenness

For calculating the evenness of species, Pielou's evenness index (*E*) was used [22].

*E* = *H*/In *S*, where *H* is the Shannon-Weiner diversity index and *S* is the total number of species in the sample.

### 2.7. Shannon-Weiner Index (*H*)

The diversity of species was calculated following the Shannon-Weiner index (*H*), which depends on the number of species present and the abundance of each species.

*H* = *Σ* *Pi* log2*Pi*, where *H* is the Shannon-Wiener index, *Pi* = *ni*/*N*, *Σ* = Sum, *ni* is the number of individuals of each species in the sample, and *N* is the total number of individuals of all species in the sample.

### 2.8. Physicochemical Parameters of Water

Water samples were collected as much as possible from the surface layer in plastic canes, avoiding unpredictable changes. The temperature, power of hydrogen ion concentration (pH), and dissolved oxygen (DO) of water were observed fortnightly on the spot. In contrast, other physicochemical parameters such as electrical conductivity (EC), turbidity, salinity, and total dissolved solids (TDS) were measured using respective digital equipment in the laboratory of Fisheries and Aquaculture, Department of Animal Sciences, Quaid-I-Azam University Islamabad.

### 2.9. Statistical Analysis

Statistically, SPSS version 26 was used for regression and correlation analysis and the relationship between variables was revealed.

## 3. Results

### 3.1. Fish Diversity of Gomal Zam Dam

In the present study, 703 fish specimens were collected from Gomal Zam Dam from October to July fortnightly bases. These specimens were identified as 18 species, 15 genera, 5 families, and 4 orders. Most of the species belonged to family Cyprinidae, the most abundant family with 14 species, whereas one species each belonged to families Siluridae, Sisoridae, Mastacembelidae, and Channidae. The observed/collected species with their classification up to genus are shown in (Table 1).

### 3.2. Distribution and Abundance of the Identified Fish Species

#### 3.2.1. *Tor putitora* (Hamilton, 1822)

*Tor putitora* was found at all three sites, Swai Nallah, Gomal village, and Gomal Khula. Highest abundance of *Tor putitora* was recorded at Gomal village (36.36%), followed by both Swai Nallah and Gomal Khula (31.81%) (Table 2). The highest monthwise abundance was recorded in December (19.31%), followed by January (15.9%), March (13.63%), July (11%), June (8%), October (5.68%), November, February, and May (7.95%). The lowest value was recorded in April (2.27%) (Table 3).

#### 3.2.2. *Cyprinion watsoni* (Day, 1872)

*Cyprinion watsoni* was recorded from all three sites. The highest abundance was recorded at Swai Nallah (43.9%), followed by Dotani village (34.14%), and the lowest value was found at Gomal Khula (21.95%) (Table 2). The highest abundance was recorded in April (26.82%), followed by May, June, and July (15%), November (12.19%), March (7.31%), and October (9.75%). However, this species was not recorded in December, January, and February (Table 3).

#### 3.2.3. *Crossocheilus diplochilus* (Heckel, 1838)

*Crossocheilus diplochilus* was recorded from all three sampling sites. The highest abundance of *Crossocheilus diplocheilus* was found at Swai Nallah (36.17%), followed by Gomal Khula (34.04%), while the minimum number was recorded from Dotani village (30%) (Table 2). Similarly, monthwise highest abundance was recorded in June (34%), followed by July (21%), of March and April (12.76%), May (10.63%), and October (8.51%). In contrast, this fish was not recorded in December, January, and February (Table 3).

#### 3.2.4. *Barilius pakistanicus* (Mirza and Sadiq 1978)

*Barilius pakistanicus* was recorded from all three sites Swai Nallah, Dotani village, and Gomal Khula. The high number of *Barilius pakistanicus* was found at Dotani village (38.14%), followed by Gomal Khula (35.05%), and the lowest number was found at Swai Nallah (Table 2). The maximum number was recorded in April (27.27%), followed by July (20%), March (18%), May (12.2%), and June (10%). While the lowest value was recorded in October (6.06%), this species was utterly absent in December, January and July (Table 3).

#### 3.2.5. *Barilius vagra* (Hamilton, 1822)

*Barilius vagra* was recorded from all sites. High abundance was recorded from Dotani village (37.93%), Swai Nallah (34.48%), and Gomal Khula (27.58%). (Table 2). The highest abundance was recorded in March (23.68%), followed by April (22.8%), July (16%), June (13%), and May (10.52%), whereas in each October and November (7.01%) but no species was found in December, January, and February (Table 3).

#### 3.2.6. *Mastacembelus armatus* (Lacepede, 1800)

*Mastacembelus armatus* was also recorded from all three sites. Its maximum number was found at Swai Nallah (57.14%), followed by Dotani village (28.57%), and the minimum number was recorded at Gomal Khula (14.28%) (Table 2), whereas the maximum number was found in July (36%), followed by June (29%) and May (21.42%), while both in October and January (7.14%). This species was absent in November, December, February, March, and April (Table 3).

#### 3.2.7. *Tor zhobensis* (Mirza, 1967)

*Tor zhobensis* was recorded merely at Dotani village and not found at Swai Nallah and Gomal Khula (Table 2). A single specimen of this species was recorded in November, utterly absent in October, December, January, February, March, April, May, June, and July (Table 3).

#### 3.2.8. *Carassius auratus* (Linnaeus, 1758)

*Carassius auratus* was recorded from all three sites. The highest abundance was found at Gomal Khula (36.58%), followed by both Swai Nallah and Dotani village (31.7%) (Table 2). The highest abundance was recorded in March and April (21.95%), followed by January (12.9%), June (10%), February (7.31%), December (7%), and July (9.75%), then in November and May (4.87%). It remained absent in October (Table 3).

#### 3.2.9. *Labeo dyocheilus* (McClelland, 1839)

*Labeo dyocheilus* was present at all three sites. The highest number was recorded from Gomal Khula (38.93%), followed by Swai Nallah (37.4%), and the lowest number was found at Dotani village (23.66%) (Table 2). Maximum abundance was found in June (19%), followed by January (15.26%) July (14%), February (12.21%), November (10.68%), December (9.92%), April (8.39%), and March (6.1%), while the lowest number was recorded in May (4.58%). However, this species was not found during October (Table 3).

#### 3.2.10. *Cyprinus carpio* (Linnaeus, 1758)

*Cyprinus carpio* was recorded from the three selected sites, but it was most abundant at Swai Nallah (43.24%), while at Gomal Khula (29.72%) and Dotani village (27.02%) it was not that abundant (Table 2). The highest percentage was recorded in July (38%), followed by December (13.51%), both in April and May (10.81%), and in March (8.1%), June (8%), and February (5.4%). The lowest number was found in November and January (2.7%), whereas absent in October (Table 3).

#### 3.2.11. *Wallago attu* (Bloch and Schneider, 1801)

*Wallago attu* was recorded only at Dotani village, and no specimen was found at Swai Nallah and Gomal Khula (Table 2). High abundance was noted in February (100%) but remained absent in October, November, December, January, March, April, May, June, and July (Table 3).

#### 3.2.12. *Cirrhinus reba* (Hamilton, 1822)

*Cirrhinus reba* was recorded from all three sites. It was most abundant at Swai Nallah (41.66%), Gomal Khula (33.33%), and least abundant at Dotani village (25%) (Table 2). The highest number was recorded in July (24%) followed by February (20%), whereas in each May and June (1%), which was followed by March (12%), June (8%), and December (4%). However, this species was not recorded in October, November, and April (Table 3).

#### 3.2.13. *Labeo diplostomus* (Heckel, 1838)

*Labeo diplostomus* was recorded from all three sites, and their highest number was recorded at Swai Nallah (35.71%), followed by each Dotani village and Gomal Khula (32.14%) (Table 2). The largest number was recorded in the month of June (30%), followed by July (26%), March (14.81%), April (11.11%), and each January and February (7.4%). In contrast, it was not found in October, November, and December (Table 3).

#### 3.2.14. *Hypophthalmichthys molitrix* (Valenciennes, 1844)

*Hypophthalmichthys molitrix* was only found at Dotani village and not seen at Swai Nallah and Gomal Khula (Table 2). A single specimen was recorded in February but remained absent during all the months (Table 3).

#### 3.2.15. *Channa marulius* (Hamilton, 1822)

*Channa marulius* was recorded from all three sites and high abundance at Gomal Khula (50%), followed by Swai Nallah (33.33%) and the lowest number at Dotani village (16.66%) (Table 2). The maximum number was found in May (33.33%), followed by December, January, February, and April (16.66%), while this species was absent in March, June, July, October and November (Table 3).

#### 3.2.16. *Ctenopharyngodon idella* (Valenciennes, 1844)

*Ctenopharyngodon idella* was found only at Gomal Khula (100%) and was absent at the other two sites (Table 2). High abundance was found during February (100%), whereas it was lacking in October, November, December, January, March, April, May, June, and July (Table 3).

#### 3.2.17. *Puntius sophore* (Hamilton, 1822)

*Puntius sophore* was recorded from all three sites. The highest number was recorded from Swai Nallah (39.28%), followed by Gomal Khula (32.14%), while the lowest number was at Dotani village (28.57%) (Table 2). Maximum abundance was recorded in May (42.85%) followed by July (25%), June (7.14%), February (3.57%), and November (21%). This species was not recorded in December, January, March, and April (Table 3).

#### 3.2.18. *Bagarius bagarius* (Hamilton, 1822)

This species was recorded at Swai Nallah and absent at Dotani village and Gomal Khula (Table 2). It was found during July but was not recorded in October, November, December, January, February, March, April, May, and June (Table 3).

The species richness, species abundance, S-Wiener index, S-diversity index, P-evenness index, and relative abundance (%R) was given in Table 4. The highest richness was found in February (10), followed by May and July (9), June (8), January (7), March, April, October, November (6), and December (4). Species abundance was high in July (125), while minimum abundance was recorded in October (28). The Shannon-Weiner index (*H*) greater value (2.37) was recorded as high during July and lower in October (1.67). The value of the Simpson diversity index (*D*) for December was (0.69) and the highest for July (0.89). The value of Pielious' evenness (*J*) was found lower in December (0.37) and higher during July and March (0.49). The relative abundance was highest (21.4) in October while lowest (5.68) in December (Table 4).

The value of species richness at Swai Nallah and Gomal Khula was recorded (14), while at Dotani village, the species richness was 13. The highest value of species abundance was calculated at Swai Nallah (249), followed by Gomal Khula (228) and Dotani village (226). The value of Shannon-Weiner (*H*) at Swai Nallah was higher (2.37) than Gomal Khula (2.29) and (2.32) at Dotani village. Similarly, the Simpson diversity index (*D*) at Dotani village was (0.88) higher than Swai Nallah (0.89) and Gomal Khula (0.88). Pielious' evenness index (*E*) was similar both at Swai Nallah and Dotani village (0.43), followed by Gomal Khula (0.42). The relative abundance was highest at Swai Nallah (0.35), while its value at Dotani village and Gomal Khula was 0.32. The % RA was also highest (35) at Swai Nallah, while its value was 32.14 at Dotani village and was 32.43 at Gomal Khula (Table 5).

### 3.3. Water Quality Parameters

The physicochemical parameters of water are shown in Table 6. The temperature, pH, dissolved oxygen, total dissolved solids, electrical conductivity, salinity, and turbidity were recorded the same at Swai Nallah, Dotani village, and Gomal Khula (Table 6).

The correlation and regression tests were conducted for finding out the relationship between temperature, pH, DO, TDS, EC, salinity, and turbidity with fish abundance Figure 2. The correlation was positive between temperature and fish abundance (*r* = 0.887). In regression analysis, the *y* value was 3.955*x* + −12.02 and *R*^2^ was 0.786. The correlation between pH and fish abundance (*r* = 0.887) was also positive, and in the regression test, the *y* value was 11.5.7*x* + −852.5 and *R*^2^ was 0.862. The correlation between DO and fish abundance (*r* = 0.967) was negative (Table 7), whereas in the regression test, the *y* value was 72.48*x* + −414.6 and value of *R*^2^ was 0.934. Similarly, the negative correlation (*r* = −0.0745) was found between TDS and fish abundance (Table 7). The regression for TDS showed that the *y* value was −0.047*x* + 97.21 and *R*^2^ was 0.005. The correlation between EC and fish abundance was negative (*r* = −0.922), and its regression showed that the *y* value was −2.575*x* + 28.56 and *R*^2^ was 0.851. The correlation between salinity and fish abundance was negative (*r* = −0.8783), whereas its regression test showed that the *y* value was −1066*x* + 637.4 and *R*^2^ was 0.771. Lastly, the correlation between turbidity and fish abundance was negative (*r* = −0.909) and its regression test showed that its *y* value was −145.8*x* + 351.7 and *R*^2^ value was 0.825 (Table 7 and Figure 2).

## 4. Discussion

The study of the fish fauna of Gomal Zam Dam was carried out from October 2018 to July 2019. A total of 18 fish species belonging to 10 families, 4 orders, and 15 genera were reported from the studied sites. Based on species richness and percentage composition, order Cypriniformes was dominant with (14 species), followed by order Siluriformes (2 species), Channiformes, and Mastacembeliformes (1 species each). The ichthyodiversity of Gomal Zam Dam consists of 5 families: Cyprinidae, Siluridae, Sisoridae, Mastacembelidae, and Channidae. The fish species we report are mainly in line with the studies conducted previously in the same region on River Zhob, [24] and water bodies of Dera Ghazi Khan region [25, 26]. The shared reported species between our and previous studies were *Cyprinion watsoni*, *Labeo dyochielus*, *Cirrihins reba*, *Barilius pakistanicus*, *Tor putitora*, *Tor zhobensis*, and *Mastacembelus armatus.* However, we did not find some previously reported species such as *Labeo rohita*, *Puntius tictto*, *Crossochielus latus*, *Aspidoparia*, *Schizocypris brucei*, *schizopygopsis stolizkae*, *Botia lohacheta*, *Glyptothorax naziri*, *Schistura kessleri*, *Schitura arifi*, and *Mastacembelus punculus*; this may be due to anthropogenic activities, illegal fishing, and particularly environmental factors because dams cause destruction of habitats of fish species and produce negative outcomes on biodiversity [27]. Human pressure, overexploitation of resources, habitat loss, and degradation of breeding grounds led to the unrecorded extinction of the restricted range species [28]. Previously, *Barilius pakistanicus* was the least abundant species from River Zhob represented by a single specimen. At the same time, we report it as one of the most abundant species forming (14.08%) of the total collection. Similarly, *Crossocheilus diplocheilus* was reported as least diverse previously, but our study represented it by 6.69%. *Cyprinion watsoni* was reported to be the most abundant species of River Zhob by both [24, 29]. In contrast, its present status in Gomal Zam Dam is 5.83%. *Barilius vagra* is the second most abundant (16.22%) species in the present study and was also reported by [29]. However, [24] did not report it previously from the regional River Zhob. These results may indicate that the favorability of the environment is proportional to fish diversity [30]. *Garra gotyla* and *Schizothorax plagiostomus* were reported from Khanozai Dam [29]; however, it was not reported from River Zhob [24], and these two species were accordingly not reported. This may be due to global warming [31] or *S. plagiostomus*, a cold-water species living at high altitudes [32]. *Tor* was also reported previously [24], and accordingly, this species was abundant in our study (12.52%). This indicates that the warm water of Gomal Zam Dam is very suitable for *T. putitora*.

In the present study, different indices were used for finding icthyodiversity, such as the Simpson diversity index, which is the probability of whether two individual fish taken from a huge community belong to a different species. This index has a value that ranges between 0 and 1. The larger the value, the more prominent will be the diversity sample [33]. In the present study, the values of the Simpson diversity index ranged from 0.88 to 0.89 at the three different sampling sites, with an overall value of 0.88 representing greater diversity for the entire region [34]. Shannon's index is the diversity (species number and evenness) comparison among different sites [35, 36]. In our study, Shannon's index value ranged from 2.29 to 2.37 in all three sampling sites, with an overall value of 2.32. The usual value of Shannon's Index range between 1.5 and 3.5, whereas elevated values indicate larger diversity [37]. Evenness indices (*E*) are used for abundance standardization [38]. Its values are considered near 0 when most individuals belong to a few species, and its values are close to 1 when species are nearly equally abundant [38]. In the present study, the evenness index ranged from 0.42 to 0.43 for three sampling sites with an overall value of 0.42. This means that most individuals belong to a few species at most of the selected sampling sites.

Physicochemical analysis of water is the prime consideration to assess its fitness to be used by aquatic animals. In the present study, water temperature ranged from 13.2-33°C to air temperature (15.8-37°C). Hasan et al. [39, 40] reported a maximum water temperature (30.5°C) in July, which is less compared to the temperature (31.8°C) we reported in June. This maximum reported temperature falls entirely in the intolerable range for the identified fish species [41]. The productivity of a water body depends on hydrogen ion concentration (pH) which indicates the acidity or alkalinity of water. pH ranges from 6.4 to 8.3 are favorable for fish growth and survival [42]. The water of Gomal Zam Dam was found to be alkaline in nature, and the pH ranged 7.3 to 8.5. In the summer months, pH values were recorded higher than in other months. This may be due to increased photosynthetic activities, which increase the nutrient concentration at higher temperatures. The solubility of drinking water can be determined by TDS because it is an important physical parameter. During the present study, the values of TDS ranged between 500 and 567 ppm. Hasan et al. [39] recorded a TDS value of 111.1–139.2 ppm while working on the physicochemical parameters of River Panjkora. The increased value of TDS indicates water pollution [43]. Dissolved oxygen is essential to all aquatic organisms and is used as an index for net biomass production [44]. The present study's range varied from 5.5 to 7.9 mg/L. Its concentration in water depends mainly upon dissolved salts, temperature, pollution load, photosynthetic activity, respiration rate, and velocity of wind [45]. The composition of the particles, presence of dissolved, suspended solids, and size and shape of particles are the various factors that affect the turbidity of water. In the present study, turbidity was measured as 0.50-2.7. Water quality measurements that can help characterize turbidity include total suspended solids, volatile suspended solids, total dissolved solids, and suspended sediment concentration.

This pioneering study reported 18 fish species dominantly of the family Cyprinidae from the three new sites of Gomal Zam Dam. The species abundance was highest from May to July and lowest from December to February. Species richness was maximum at Swai Nallah and Gomal Khula, while it was minimum at Dotani village. We recommend further studies to explore other undiscovered water bodies of Pakistan for ichthyofaunal diversity. Moreover, we recommend DNA-based identification for taxonomic and evolutionary allocation of the fish.

## Figures and Tables

**Figure 1:** Map and location of Gomal Zam Dam and its tributaries. The three sampling sites were shown in the map. The map was cropped from Google Map and was edited accordingly.

**Figure 2:** The regression between water quality parameters and fish abundance. Values for each parameter (a–g) are shown in *x*-axis while fish abundance is shown in *y*-axis, respectively.

**Table 1:** Fish species reported in this study from Gomal Zam Dam.

Family	Genus	Species
Mastacembelidae	Mastacembelus	*M. armatus*
Channidae	Channa	*C. marulius*
Siluridae	Wallago	*W. attu*
Sisordiae	Bagarius	*B. bagarius*
Cyprinidae	Tor	*T. zhobensis,*
		*T. putitora*
**//**	Barilus	*B. pakistanicus,*
		*B. vagra*
**//**	Labeo	*dyochielus, diplostomus*
		*L. diplostomus*
**//**	Cirrihinus	*C. reba*
**//**	Hyphophthalmicthys	*H. molitrix*
**//**	Ctenophyringodon	*C. idella*
**//**	Puntius	*P. sophore*
**//**	Crossochielus	*C. diplochielus*
**//**	Carassius	*C. auratus*

**Table 2:** Sitewise fish species recorded during the study from Gomal Zam Dam. The conservation status of each species was given according to Bibi et al. [23] and IUCN 2021-3 [46].

Species	Conservation status	Swai Nallah, *n* (%)	Dotani village, *n* (%)	Gomal Khula, *n* (%)	Ab	RA	%RA
*T. putitora*	Endangered	28 (31.81)	32 (36.36)	28 (31.81)	88	0.13	12.52
*C. watsoni*	Least concern	18 (43.90)	14 (34.14)	9 (21.95)	41	0.06	5.83
*C. diplocheilus*	Least concern	17 (36.17)	14 (29.78)	16 (34.04)	47	0.07	6.69
*B. pakistanicus*	Not evaluated	26 (26.80)	37 (38.14)	34 (35.05)	97	0.14	13.80
*B. vagra*	Least concern	40 (34.48)	44 (37.93)	32 (27.58)	116	0.17	16.50
*M. armatus*	Least concern	8 (57.14)	4 (28.57)	2 (14.28)	14	0.02	1.99
*T. zhobensis*	Not evaluated	0 (0)	1 (100)	0 (0)	1	0.00	0.14
*C. auratus*	Least concern	13 (31.70)	13 (31.70)	15 (36.58)	41	0.06	5.83
*L. dycheilus*	Least concern	49 (37.40)	31 (23.66)	51 (38.93)	131	0.19	18.63
*C. carpio*	Vulnerable	16 (43.24)	10 (27.02)	11 (29.72)	37	0.05	5.26
*W. attu*	Near threatened	0 (0)	1 (100)	0 (0)	1	0.00	0.14
*C. reba*	Least concern	10 (41.66)	6 (25)	8 (33.33)	24	0.03	3.41
*L. diplostomus*	Least concern	10 (35.71)	9 (32.14)	9 (32.14)	28	0.04	3.98
*H. molitrix*	Near threatened	0 (0)	1 (100)	0 (0)	1	0.00	0.14
*C. marulius*	Least concern	2 (33.33)	1 (16.66)	3 (50)	6	0.01	0.85
*C. idella*	Not evaluated	0 (0)	0 (0)	1 (100)	1	0.00	0.14
*P. sophore*	Least concern	11 (39.28)	8 (28.57)	9 (32.14)	28	0.04	3.98
*B. bagarius*	Near threatened	1 (100)	0 (0)	0 (0)	1	0.00	0.14
Total		249	226	228	703	1.00	100.0

**Table 3:** Monthwise abundance of fish species recorded during the study from Gomal Zam Dam.

Species	Oct. *n* (%)	Nov. *n* (%)	Dec. *n* (%)	Jan. *n* (%)	Feb. *n* (%)	Mar. *n* (%)	Apr. *n* (%)	May *n* (%)	June *n* (%)	July *n* (%)	Ab	RA	%RA
*T. putitora*	5 (5.7)	7 (7.2)	17 (19.3)	14 (15.9)	7 (7.)	12 (13.6)	2 (2.3)	7 (7.9)	7 (7.9)	10 (1.36)	88	0.13	12.5
*C. watsoni*	4 (9.8)	5 (12.2)	0 (0)	0 (0)	0 (0)	3 (7.3)	11 (26.8)	6 (14.6)	6 (14.6)	6 (14.6)	41	0.06	5.8
*C.diplocheilus*	4 (8.5)	0 (0)	0 (0)	0 (0)	0 (0)	6 (12.8)	6 (12.8)	5 (10.6)	16 (34.0)	10 (21.27)	47	0.07	6.7
*B.pakistanicus*	6 (6.1)	4 (4.0)	0 (0)	0 (0)	0 (0)	18 (18.2)	27 (27.3)	12 (12.1)	12 (12.1)	20 (20.2)	99	0.14	14.1
*Bariliusvagra*	8 (7.0)	8 (7.0)	0 (0)	0 (0)	0 (0)	27 (23.7)	26 (22.8)	12 (10.5)	15 (13.2)	18 (15.9)	114	0.16	16.2
*M. armatus*	1 (7.1)	0 (0)	0 (0)	1 (7.1)	0 (0)	0 (0)	0 (0)	3 (21.42)	4 (28.6)	5 (35.7)	14	0.02	1.9
*T.zhobensis*	0 (0)	1 (100)	0 (0)	0 (0)	0 (0)	0 (0)	0 (0)	0 (0)	0 (0)	0 (0)	1	0.00	0.1
*C. auratus*	0 (0)	2 (4.9)	3 (7.3)	5 (12.2)	4 (9.7)	9 (21.9)	9 (21.9)	2 (4.9)	4 (9.7)	3 (7.3)	41	0.06	5.8
*L. dycheilus*	0 (0)	14 (10.7)	13 (9.9)	20 (15.3)	16 (12.2)	8 (6.1)	11 (8.4)	6 (4.6)	25 (19.1)	18 (13.7)	131	0.19	18.63
*C. carpio*	0 (0)	1 (2.7)	5 (13.5)	1 (2.70)	2 (5.4)	3 (8.1)	4 (10.8)	4 (10.8)	3 (8.1)	14 (37.8)	37	0.05	5.26
*W. attu*	0 (0)	0 (0)	0 (0)	0 (0)	1 (100)	0 (0)	0 (0)	0 (0)	0 (0)	0 (0)	1	0.00	0.14
*C. reba*	0 (0)	0 (0)	1 (4)	2 (8)	5 (20)	3 (12)	0 (0)	4 (16)	4 (16)	6 (24)	25	0.04	3.56
*L. diplostomus*	0 (0)	0 (0)	0 (0)	2 (7.4)	2 (7.4)	4 (14.8)	3 (11.1)	1 (3.7)	8 (29.62)	7 (25.92)	27	0.04	3.84
*H. molitrix*	0 (0)	0 (0)	0 (0)	0 (0)	1 (100)	0 (0)	0 (0)	0 (0)	0 (0)	0 (0)	1	0.00	0.14
*C. marulius*	0 (0)	0 (0)	1 (16.7)	1 (16.7)	1 (16.7)	0 (0)	1 (16.7)	2 (33.3)	0 (0)	0 (0)	6	0.01	0.85
*C. idella*	0 (0)	0 (0)	0 (0)	0 (0)	1 (100)	0 (0)	0 (0)	0 (0)	0 (0)	0 (0)	1	0.00	0.14
*P. spore*	0 (0)	1 (3.6)	0 (0)	0 (0)	2 (7.1)	0 (0)	0 (0)	12 (42.8)	6 (21.4)	7 (25)	28	0.04	3.98
*B. bagarius*	0 (0)	0 (0)	0 (0)	0 (0)	0 (0)	0 (0)	0 (0)	0 (0)	0 (0)	1 (100)	1	0.00	0.14
Grand total	28	43	40	46	42	93	100	76	110	125	703	1	100

**Table 4:** Different ichthyodiversity-related parameter recorded monthwise in the study from Gomal Zam Dam.

Parameters	Months									
	Oct.	Nov.	Dec.	Jan.	Feb.	Mar.	Apr.	May	June	July
Species richness	6	6	4	7	10	6	6	9	8	9
Species abundance	28	43	40	46	42	93	100	76	110	125
S-Wiener index	1.67	1.85	1.37	1.49	1.93	1.92	1.93	2.36	2.27	2.37
*S*-diversity index	0.8	0.81	0.69	0.7	0.79	0.84	0.82	0.89	0.88	0.89
*P*-evenness index	0.5	0.49	0.37	0.39	0.52	0.49	0.42	0.52	0.48	0.49
Relative abundance	0.21	0.06	0.05	0.06	0.05	0.013	0.14	0.1	0.15	0.17
%RA	21.4	6.11	5.68	6.54	5.97	13.22	14.22	10.81	15.64	17.78

**Table 5:** Different ichthyodiversity-related parameter recorded sitewise in the study from Gomal Zam Dam.

Parameters	Study sites		
	Swai Nallah	Dotani village	Gomal Khula
Species richness	14	13	14
Species abundance	249	226	228
Shannon-Wiener index	2.37	2.32	2.29
Simpson diversity index	0.89	0.88	0.88
Pielious' evenness index	0.43	0.43	0.42
Relative abundance	0.35	0.32	0.32
%R A	35	32.14	32.43

**Table 6:** Mean ± SD of physicochemical parameters from the studied sites of Gomal Zam Dam.

Variables	Units	Swai Nallah	Dotani village	Gomal Khula
Temp	°C	20.81 ± 7.78	20.13 ± 6.99	20.49 ± 7.42
pH	pH unit	7.97 ± 0.26	7.73 ± 0.27	7.73 ± 0.27
DO	mg/L	6.53 ± 0.53	6.65 ± 0.98	6.78 ± 0.82
TDS	mg/L	518.9 ± 12.36	545.10 ± 13.11	519.10 ± 12.36
EC	*μ*S/cm	1074.6 ± 15.04	1080.60 ± 17.73	1075.50 ± 25.55
Salinity	mg/L	0.52 ± 0.03	0.53 ± 0.03	0.53 ± 0.03
Turbidity	mg/L	2.04 ± 0.26	2.00 ± 0.29	2.07 ± 0.35

**Table 7:** Correlation analysis of water quality parameters versus fish abundance.

Variable	Correlation values (*r*)	Correlation status
Temp vs. fish abundance	0.887	Positive
PH vs. fish abundance	0.86	Positive
DO vs. fish abundance	0.96	Positive
TDS vs. fish abundance	-0.074	Negative
EC vs. fish abundance	-0.92	Negative
Salinity vs. fish abundance	-0.87	Negative
Turbidity vs. fish abundance	-0.90	Negative

## Data Availability

The data was generated from record of the survey conducted during the field visit on hard paper; therefore, it cannot be converted into soft form to be available online.
